The article "Bone Mechanoregulation Allows Subject-Specific Load Estimation Based on Time-Lapsed Micro-CT and HR-pQCT in Vivo" was published in 2021. Journal: Front Bioeng Biotechnol.

# Bone Mechanoregulation Allows Subject-Specific Load Estimation Based on Time-Lapsed Micro-CT and HR-pQCT *in Vivo*

**DOI:** 10.3389/fbioe.2021.677985

**Published:** 2021-06-25

**Authors:** Matthias Walle, Francisco C. Marques, Nicholas Ohs, Michael Blauth, Ralph Müller, Caitlyn J. Collins

**Affiliations:** ^1^Institute for Biomechanics, ETH Zurich, Zurich, Switzerland; ^2^Department for Trauma Surgery, Innsbruck University Hospital, Innsbruck, Austria

**Keywords:** bone loading estimation, mechanoregulation, finite element analysis, bone remodelling, human distal radius, mouse caudal vertebra

## Abstract

Patients at high risk of fracture due to metabolic diseases frequently undergo long-term antiresorptive therapy. However, in some patients, treatment is unsuccessful in preventing fractures or causes severe adverse health outcomes. Understanding load-driven bone remodelling, i.e., mechanoregulation, is critical to understand which patients are at risk for progressive bone degeneration and may enable better patient selection or adaptive therapeutic intervention strategies. Bone microarchitecture assessment using high-resolution peripheral quantitative computed tomography (HR-pQCT) combined with computed mechanical loads has successfully been used to investigate bone mechanoregulation at the trabecular level. To obtain the required mechanical loads that induce local variances in mechanical strain and cause bone remodelling, estimation of physiological loading is essential. Current models homogenise strain patterns throughout the bone to estimate load distribution *in vivo*, assuming that the bone structure is in biomechanical homoeostasis. Yet, this assumption may be flawed for investigating alterations in bone mechanoregulation. By further utilising available spatiotemporal information of time-lapsed bone imaging studies, we developed a mechanoregulation-based load estimation (MR) algorithm. MR calculates organ-scale loads by scaling and superimposing a set of predefined independent unit loads to optimise measured bone formation in high-, quiescence in medium-, and resorption in low-strain regions. We benchmarked our algorithm against a previously published load history (LH) algorithm using synthetic data, micro-CT images of murine vertebrae under defined experimental *in vivo* loadings, and HR-pQCT images from seven patients. Our algorithm consistently outperformed LH in all three datasets. *In silico*-generated time evolutions of distal radius geometries (*n* = 5) indicated significantly higher sensitivity, specificity, and accuracy for MR than LH (*p* < 0.01). This increased performance led to substantially better discrimination between physiological and extra-physiological loading in mice (*n* = 8). Moreover, a significantly (*p* < 0.01) higher association between remodelling events and computed local mechanical signals was found using MR [correct classification rate (CCR) = 0.42] than LH (CCR = 0.38) to estimate human distal radius loading. Future applications of MR may enable clinicians to link subtle changes in bone strength to changes in day-to-day loading, identifying weak spots in the bone microstructure for local intervention and personalised treatment approaches.

The article "Bone Mechanoregulation Allows Subject-Specific Load Estimation Based on Time-Lapsed Micro-CT and HR-pQCT in Vivo" was published in 2021. Journal: Front Bioeng Biotechnol.

## Introduction

Considerable patient variability in bone structure, strength, and day-to-day external mechanical load poses a severe problem in the clinical assessment and treatment of metabolic bone diseases such as osteoporosis. Diagnosis and bone strength assessment rely heavily on radiographic measures of bone mineral density (BMD). However, sources of error in BMD measurements, i.e., intra- and interpatient variability, make it challenging to attribute measured BMD changes to the actual biological change (Nguyen et al., 1997). Accordingly, the sensitivity and specificity of predicting individual patient’s risk for fracture are low (Trémollieres et al., 2010; Cervinka et al., 2017), especially at the hip where falls play a major role. As a consequence, patients may receive treatment, although only a minority would have suffered from a bone fracture. Although these medications are well-tolerated and safe during large-scale clinical trials, anti-resorptive therapies can result in rare and severe adverse events, including osteonecrosis, hypocalcaemia, and thromboembolism (Chen and Sambrook, 2012). Moreover, current diagnostic approaches fail to identify the specific weak spots in the bone. Therefore, they do not estimate where and how fractures will occur and how a local intervention could prevent them (Schultz and Wolf, 2019).

High-resolution peripheral quantitative computed tomography (HR-pQCT), an emerging diagnostic modality of the peripheral skeleton, allows assessing three-dimensional (3D) bone structure and strength at the trabecular level (MacNeil and Boyd, 2007; Melton et al., 2007; Boutroy et al., 2008; Kazakia et al., 2008; Burghardt et al., 2010; Seeman et al., 2010; MacDonald et al., 2011). More recently, complementary methods have been proposed to computationally monitor 3D bone microstructure changes over time (time-lapse) and calculate local mechanical loading using micro-finite element (micro-FE) analysis. This has been demonstrated in mice (Schulte et al., 2013; né Betts et al., 2020; Malhotra et al., 2021) and patients (Christen et al., 2014; Mancuso and Troy, 2020) at such high spatial resolution that cellular behaviour—in the form of bone remodelling sites—can be studied and the corresponding mechanical loading can be calculated. Subsequently, these methods can be used to investigate bone’s underlying mechanoregulated remodelling process, which may be the key to the development of patient-specific therapeutic or pharmacological interventions for various bone diseases.

The article "Bone Mechanoregulation Allows Subject-Specific Load Estimation Based on Time-Lapsed Micro-CT and HR-pQCT in Vivo" was published in 2021. Journal: Front Bioeng Biotechnol.

Typically, when investigating bone mechanoregulation under controlled experimental conditions, micro-FE models disregard subject-specific variations in external loading conditions using simplified uniaxial compressive displacement boundary conditions (SC) (Schulte et al., 2013; Mancuso and Troy, 2020; né Betts et al., 2020; Malhotra et al., 2021). However, when investigating mechanoregulation in patients, variations in day-to-day external loading are more substantial due to habitual differences and patient-specific variability in the musculoskeletal system’s performance. Distinctive tensile forces and moments are applied to joints on a routine basis to stabilise under gravitational and other external loads and create unique loading patterns (Watkins, 2009). Consequently, to investigate mechanoregulation under day-to-day loading in a personalised medicine approach, patient-specific physiological loading patterns and boundary conditions need to be estimated (Galibarov et al., 2010; Yosibash et al., 2020).

In an effort to quantify *in vivo* loading patterns using biomechanical models, several load estimation algorithms have been developed. Artificial neural network-based approaches have been proposed (Garijo et al., 2014, 2017; Mouloodi et al., 2020) but lack interpretability, which is critical for moving to diagnostic use in patients to guide local therapeutic interventions. As a result, an algebraic method introduced by Christen et al. (2012) has been widely implemented to approximate the internal load history based on bone morphology (Christen et al., 2014; Badilatti et al., 2017; Synek et al., 2019; Cheong et al., 2020; né Betts et al., 2020). This algorithm superimposes and scales a finite number of loading cases until a target tissue load of homogeneous strains is found. Christen et al. (2012) demonstrated the capabilities of such a reverse-engineering approach using an extra-physiological tail-loading animal model, predicting the applied compressive loading in mouse caudal vertebra. However, the remaining signal inhomogeneity remained high, ranging between 20% and 67%, indicating that no homogeneous tissue load could be found (Christen et al., 2012). This suggests that only part of the bone structure may be load adapted. The actual *in vivo* load distribution might differ systematically from the homogeneous assumption in humans (Christen et al., 2016; Johnson and Troy, 2018) and mice (Christen et al., 2012). By modelling homogenised strain patterns, the conventional algorithm may reduce mechanical signal inhomogeneities that have been recognised as drivers for the mechanoregulated remodelling process in bone (Frost, 1987, 2003). Thus, this model’s assumptions may not be optimal and do not fully utilise all available information in time-lapsed data of longitudinal bone imaging studies.

The article "Bone Mechanoregulation Allows Subject-Specific Load Estimation Based on Time-Lapsed Micro-CT and HR-pQCT in Vivo" was published in 2021. Journal: Front Bioeng Biotechnol.

This study had two goals. First, to derive an *in silico*-validated, robust, and specific method to estimate *in vivo* loading. Second, to apply this algorithm to examine *in vivo* mechanoregulation (Schulte et al., 2013) in humans and mice. We hypothesised that by extracting bone remodelling sites from time-lapsed imaging data, the relationship between bone formation in high-strain regions, quiescence in medium-strain regions, and resorption in low-strain regions could be used in a reverse-engineering optimisation approach to determine organ-level loads. We verified our mechanoregulated approach (MR) using three unique datasets and benchmarked it with an existing load history (LH) algorithm (Christen et al., 2012). First, to calculate sensitivity, specificity, and accuracy, MR and LH algorithms were applied to synthetic remodelling data derived from HR-pQCT images (Badilatti et al., 2016; Ohs et al., 2020a). Second, to test whether the algorithms are capable of predicting the loading conditions in a controlled experimental setup, both algorithms were applied to micro-CT scans of two groups of mice that had their caudal vertebra either loaded (8 N) or sham loaded (0 N) from a previous study (Scheuren et al., 2020b). Third, to assess the method’s fidelity in patients, MR and LH algorithms were applied to time-lapsed HR-pQCT scans and compared to patient-specific handgrip force measured using a dynamometer. Finally, to quantify the association between bone remodelling and mechanical stimulus, we derived a correct classification rate (CCR) (né Betts et al., 2020).

## Materials and Methods

### Human HR-pQCT Images *in vivo*

HR-pQCT images (XtremeCT II, 60.7 μm voxel size, 68 kV, 1,470 μA, integration time of 43 ms) were acquired from the database of a prior Innsbruck Medical University fracture study (Atkins et al., 2021). Patients gave informed consent and participated in an examination approved by the Medical University of Innsbruck Ethics Committee (UN 0374344/4.31). For each patient, scans of the intact contralateral radius were taken at six time points (1, 3, 5, 13, 26, and 52 weeks) post-fracture, 9 mm proximal to the endplate of the distal radius (Figure 1). As a functional indicator of daily mechanical load, handgrip strength was measured at 3, 6, and 12 months post-fracture using a hydraulic handgrip dynamometer. Grip strength was taken in a seated position with the elbow bent 90 degrees in flexion, measured three times and averaged. Measurements were recorded in kilograms and converted to Newtons (1 kg ↔ 9.81 N). Images were graded by two skilled operators using a standard visual grading score (VSG) ranging from 1 (no visible motion artefacts) to 5 (major horizontal streaks) (Whittier et al., 2020). Distal radius images of seven patients (three males, four females) were included in the study by applying the following inclusion criteria. Only males or premenopausal female patients without a fracture history of their non-dominant left distal radius were included. Only patients for whom all scans met a minimum VSG of 3 (some artefacts) and a VGS of less than or equal to 2 (very slight artefacts) in four out of the six total follow-up scans were included. The median age of the included patients was 33 years and ranged between 27 and 65 years.

The article "Bone Mechanoregulation Allows Subject-Specific Load Estimation Based on Time-Lapsed Micro-CT and HR-pQCT in Vivo" was published in 2021. Journal: Front Bioeng Biotechnol.

**FIGURE 1:** Representative fluoroscopic images of *in vivo* scanning sites. The C6 mouse caudal vertebra (dashed box, left) was scanned by micro-CT. Black lines indicate sites of loading pins in the C5 (clamped) and C7 (loaded) vertebra. A representative loading scenario is indicated below for physiologically loaded (phys.) and extra-physiologically loaded (loaded) groups throughout the study (t_0_–t_4_). The human distal radius (dashed box, right) was scanned using high-resolution peripheral quantitative computed tomography (HR-pQCT; Xtreme CT II). Annotations indicate the manufacturer’s recommended scanning site, 9 mm proximal to the reference line, and the arrows represent the line of action of the joint forces on the radius as a result of physiological loading. The box below indicates representative loading throughout appointments t_0_–t_5_.

### Murine Micro-CT Images *in vivo*

Micro-CT images (vivaCT 40, 10.5 μm voxel size, 55 KVp, 145 μA, integration time of 350 ms, 500 projections) were acquired from a previously published mouse tail loading study (Scheuren et al., 2020b). Two groups (*n* = 8, each) of 15-week-old female C57BL/6J strain mice were scanned at the sixth caudal vertebra (CV6) at weekly intervals for 5 weeks. The sixth caudal vertebra of the animals in the loaded group was subject to mechanical loading through stainless steel pins inserted into the adjacent vertebrae (Figure 1). Compressive loading was applied three times per week for 5 min at 10 Hz and 8 N. Animals in the control group were subject to sham loading (0 N) (see Scheuren et al., 2020b).

The article "Bone Mechanoregulation Allows Subject-Specific Load Estimation Based on Time-Lapsed Micro-CT and HR-pQCT in Vivo" was published in 2021. Journal: Front Bioeng Biotechnol.

### Image Processing

After rigid image registration (Schulte et al., 2014), distal radius images were upscaled to 30.5 μm (Ohs et al., 2020a), and caudal vertebra images were kept at 10.5 μm native resolution. Images were Gauss filtered to reduce noise (sigma 1.2, support 1). Human distal radius and mouse vertebra scans were binarised using a threshold of 320 and 580 mg/cm^3^, respectively (Hosseini et al., 2017; Scheuren et al., 2020a). Trabecular regions were automatically contoured from binarised images. For the human distal radius images, an approach described by Ohs et al. (2020b) was used; for the mouse vertebra images, a method described by Kohler et al. (2007) was used. FE meshes were generated by converting all voxels to 8 node hexahedral elements and assigning a Poisson’s ratio of 0.3 as well as Young’s modulus of 6.8 GPa for the human distal radius (Christen et al., 2013) and 14.8 GPa (Webster et al., 2008) for the mouse vertebra. Remaining interior voxels located within the bone cavity were assigned a value of 2 MPa and a Poisson’s ratio of 0.3 (Webster et al., 2008). For the mouse caudal vertebra, intervertebral discs with a Young’s modulus of 14.8 GPa were approximated and added to the proximal and distal ends of the vertebra (Webster et al., 2008; Schulte et al., 2013).

### Micro-Finite Element Analysis

Axial and shear forces were applied to the target tissue’s distal and proximal surfaces using a 1% displacement boundary condition. Torsion and bending moments were applied, centred around their corresponding axis, with a 1-degree displacement. The point of reference was the centre of the minimal bounding box enclosing the bone geometry. Six loading directions were defined: compressive force in the axial direction (C, *Z*-axis), lateral shear force (SX, *X*-axis), dorsal shear force (SY, *Y*-axis), axial moment around the long axis (MZ, *Z*-axis), lateral bending moment (BX, *X*-axis), and dorsal bending moment (BY, *Y*-axis). Models averaged 20 million elements for the mouse vertebrae and 380 million elements for the distal radii at the upscaled resolution (30.5 μm voxel size). Linear FE calculations were carried out using ParOsol (Flaig and Arbenz, 2011) at the Swiss National Supercomputing Centre (CSCS, Lugano, Switzerland). Using 128 CPUs, the solver converged in under 10 min for distal radii and under 1 min for caudal vertebrae. Strain energy density (SED) was used as a mechanical signal for bone remodelling. Unit load cases were derived by rescaling applied force magnitudes to 1 N, moment magnitudes to 1 Nmm, and resulting SED distributions accordingly (Christen et al., 2012). Three multiaxial loads were defined using a method of scaling and superimposing unit load cases modelling the aggregated effect of physiological load over time: combined compression and shear (CS = 0.5 C + 0.25 SX + 0.25 SY), combined compression and bending (CB = 0.5 C + 0.25 BX + 0.25 BY), and a combined 6-degree freedom load (6DoF) with equal proportions of load in all six uniaxial directions.

The article "Bone Mechanoregulation Allows Subject-Specific Load Estimation Based on Time-Lapsed Micro-CT and HR-pQCT in Vivo" was published in 2021. Journal: Front Bioeng Biotechnol.

### Mechanoregulation-Based Load Estimation

The mechanoregulation-based load estimation (MR) was performed in two steps and followed established mechanoregulation principles (Wolff, 1892). Using a two-step procedure instead of additional constraints to the optimiser reduced computational cost and led to faster convergence of the optimiser within 2,000 iterations in under a minute. The algorithm operated on the bone surface S(x), which was defined as the interface between the bone and the background using a 3D von Neumann neighbourhood with a radius of 1 voxel. New bone was presumed to be formed in high mechanical signal regions, quiescent in regions of medium mechanical signal, and resorbed in regions of low mechanical signal (Figure 2). Regions of formation RV_f_, quiescence RV_q_, and resorption RV_r_ were calculated by overlaying two subsequent binary images aligned using rigid registration. Each surface voxel was assigned a rank rg_*RS*_ according to its remodelling event (resorption = 1, quiescence = 2, and formation = 3). Accordingly, an ordinal definition of the mechanical signal rg_SED_ was specified with increasing rank for increasing signal magnitude. Equal observations were assigned the mean rank for their positions. The monotonic relationship between rg_RS_ and rg_SED_ represents a mechanoregulated behaviour between surface remodelling events and mechanical signal.

**FIGURE 2:** Overview of the mechanoregulation-based load estimation (MR) algorithm and morphology-based load history (LH) algorithm. (Top left) *In vivo* loading is assessed by MR between two consecutive images, outlining the algorithm’s field of view (FOV). By overlaying registered longitudinal images, remodelling regions are identified to find a loading scenario maximising the correlation between formation (F) in regions of high strain, quiescence (Q) in regions of medium strain, and resorption (R) in regions of low strain. (Bottom left) In comparison, load history (LH) estimates the complete *in vivo* load history with no option to limit its FOV and targets a homogeneous strain distribution of medium strain (0.02 MPa). (Center) For the optimisation in both algorithms, micro-finite element (FE) models are created covering all physiologically possible loading directions. During the optimisation, unit loads are scaled until the optimisation target is achieved, providing (Top right) individual load components (i.e., forces and moments) as well as (Bottom right) a combined load distribution.

The article "Bone Mechanoregulation Allows Subject-Specific Load Estimation Based on Time-Lapsed Micro-CT and HR-pQCT in Vivo" was published in 2021. Journal: Front Bioeng Biotechnol.

In the first optimisation step, Spearman’s rank-order correlation between rg_*RS*_ and rg_SED_ was maximised by scaling a set of previously defined unit load cases U_(i,unit)_(x) with load composition factors c_i_ (with c_i_ ∈ [0, 1]), where U_(i,unit)_(x) is the SED distribution due to unit load i on the bone surface S(x). The superimposed unit loads defined a potential compounded mechanical stimulus with known unit load proportions within each iteration. A gradient-free Nelder–Mead method with a tolerance of 10^–4^ was used to optimise the following resulting equivalent minimisation objective function r. A non-negative linear least-squares solution of homogeneous tissue loading (*k* = 0.02 MPa) was used to initialise the optimiser.

$$\begin{array}{c} \min r\left(c_{i}\right)=-corr\left(rg_{SED}\left(\sum_{i=0}^{n}c_{i}*U_{i,unit}\left(x\right)\right),rg_{RS}\right) \end{array}$$

The resulting load composition c_i_ determined the best combination of unit loads (C, SX, SY, MZ, BX, and BY) to associate bone formation in regions of high, quiescence in areas of medium, and resorption in regions of low signal for two subsequent images. However, no assumptions on the magnitude of the mechanical signal were made. To derive the final mechanical load, a second optimisation procedure matching the compounded signal with the bone’s overall remodelling response was performed on the entire bone volume. Bone formation rate (BFR), bone resorption rate (BRR), and net remodelling response (NRR = BFR - BRR) were calculated from the registered binary images (Lambers et al., 2011; Schulte et al., 2011). To calculate NRR_SED_ as predicted by the mechanical signal, we defined a ternary classifier function f_j_ considering two thresholds for sites of formation T_f_ and sites of resorption T_r_ according to né Betts et al. (2020). The thresholds T_f_ = 0.0204 MPa and T_r_ = 0.0196 MPa were chosen based on average bone loading values of 0.02 MPa from previous studies (Christen et al., 2012, 2013). To observe both, formation and resorption, in the simulations, a narrow 4%-wide lazy zone was implemented. At each iteration, NRR_SED_ was calculated by scaling the compounded mechanical signal using a second scaling factor r, and the prediction of the classifier function f_j_ (r *Σc_i_ * U_*i,unit*_[x]) within was used in the current study. A gradient-free Nelder–Mead method with a tolerance of 10^–4^ was used to minimise the difference between NRR_SED_ and NRR_*GT*_ using the following objective function k(r).

$$\begin{array}{c} \min k\left(r\right)=\left|{\mathrm{NRR}}_{SED}\left(r\right)-NRR_{GT}\right| \end{array}$$

For consistency with Christen et al. (2013), scaling factors c_i_ and r were incorporated into a single scaling factor s_i_ = r * c_i_, which combines magnitude and number of load cycles applied over time. Assuming each load case acted equally long over time and was applied sequentially, loading magnitude α_i_ was calculated as α_i_ = √(6 * s_i_) for the six applied unit load cases.

The article "Bone Mechanoregulation Allows Subject-Specific Load Estimation Based on Time-Lapsed Micro-CT and HR-pQCT in Vivo" was published in 2021. Journal: Front Bioeng Biotechnol.

### Morphology-Based Load History Estimation

Following a previously published approach (Christen et al., 2013), we implemented an LH algorithm. Unit load cases were scaled using load composition factors s_i_ until the most homogeneous distribution is found (*k* = 0.02 MPa) (Figure 2). Scaling factors s_i_ were calculated using a non-negative linear least-squares optimisation technique, and load magnitudes α_i_ were calculated as previously described. Furthermore, a calibrated version of LH was implemented (cal. LH). In its native implementation, LH evaluates the load history before the imaging time point. In longitudinal studies, physiological loading during the study may change compared to loading before the study. To reduce this initial bias from prior loading, the scaling factors estimated by LH α_*i,t–1*_ from the previous baseline image were subtracted from the estimated scaling factors α_*i,t*_ of the current timestep. To derive applied loading magnitudes from cal. LH, linear regressions between cal. LH and the applied load were calculated.

### Study Design

First, *in silico* geometries were derived from HR-pQCT images and adapted using a model of load-adaptive remodelling. Receiver operating characteristics (ROCs) were used to compare simulated to estimated loads and calculate sensitivity, specificity, and accuracy. Second, MR and LH algorithms were applied to longitudinal micro-CT scans of the sixth caudal vertebra in mice loaded extra-physiologically and sham-loaded controls. Root mean square error (RMSE) between experimentally derived and estimated SED was calculated. Third, MR and LH algorithms were applied to longitudinal HR-pQCT scans of the distal radius from patients whose handgrip force was measured using a dynamometer. Pearson’s correlation (R) between predicted load and grip strength was calculated, assessing the method’s fidelity. Finally, bone mechanoregulation was investigated for all three image data sets using MR, LH, and simplified compression loads as input for the boundary conditions. Conditional probabilities (CP) were calculated, associating surface remodelling events with SED levels. To quantify the proportion of mechanoregulated remodelling, a maximum CCR was used.

The article "Bone Mechanoregulation Allows Subject-Specific Load Estimation Based on Time-Lapsed Micro-CT and HR-pQCT in Vivo" was published in 2021. Journal: Front Bioeng Biotechnol.

#### Generation of Adapted Bone Geometries *in silico*

For the *in silico* experiments, five patients (four females, one male) with VGS lower than 2 were randomly selected from the initial patient cohort due to the high computational cost of the remodelling simulation. Geometries derived from baseline HR-pQCT scans were adapted toward previously defined uniaxial (C, SX, SY, MZ, BX, and BY) and multiaxial (CS, CB, and 6DoF) loads using a modified advection-based remodelling algorithm (Badilatti et al., 2016; Ohs et al., 2020a). In short, a regularised density that matched binary bone volume fraction (BV/TV) while preserving greyscale value on the bone surface was converted to Young’s modulus using a linear relationship (Mulder et al., 2007) and used as input for the remodelling algorithm (Ohs et al., 2020a). The advection-based remodelling process, as described in Figure 3, was limited to the trabecular region and performed for each of the nine *in silico* loading experiments for 40 remodelling steps. SED and applied force magnitudes derived from micro-FE analyses were rescaled to target sample-specific homoeostatic remodelling with comparable amounts (< 2% difference) of bone formation and resorption. Changes in voxel-by-voxel intensity between subsequent remodelling steps were quantified using Pearson correlation. From each simulation, six time points were subsampled by increasing the time interval between selected time points until a Pearson correlation of at least 0.95 was reached between subsequent scans. This subsampling procedure was performed to model a change in tissue volume comparable to our *in vivo* HR-pQCT data.

**FIGURE 3:** Schematic workflow to derive bone geometries from advection-based remodelling simulations. Input, greyscale high-resolution peripheral quantitative computed tomography (HR-pQCT) images of the distal radius were first Gauss-filtered and regularised before finite element modelling. Strain energy density (SED) was derived from a linear finite element analysis (FEA), and cell sensing was mimicked through mechanical signal dilation with a fixed radius of 50 μm. Tissue was remodelled using a SED-dependent velocity of ± 8,000 μm/year/MPa and a maximum velocity of ± 12 μm/month in regions where SED exceeded or fell short of the average tissue load (0.02 MPa) by ± 2%, and the growth direction was simulated normal to the bone surface. An advection step performed the surface movement, either resorption (R, purple) or formation (F, yellow), and a remodelled output regularised image was derived. Quiescence (Q) was modelled as no surface movement. This process repeats with the regularised output image as input for the next iteration (n).

The article "Bone Mechanoregulation Allows Subject-Specific Load Estimation Based on Time-Lapsed Micro-CT and HR-pQCT in Vivo" was published in 2021. Journal: Front Bioeng Biotechnol.

#### Sensitivity, Specificity, and Accuracy *in silico*

A multiclass ROC averaging approach was used to assess the accuracy of the *in silico* load estimation. For moments (Nmm), a corresponding torque force (N) applied at the minimum bounding box and about the point of reference was calculated to allow comparison between loadings. Specifically, the torque lever arm was half the stack height for bending; for torsion, the torque lever arm was half the dorsal length of the minimum bounding box of the distal radius geometry. The Euclidean distances between the estimated and all possibly applied force vectors [N] were calculated. A percentage error was calculated by dividing the Euclidean distance by the applied force as a scalar error quantification. The multiclass prediction of all nine *in silico* loading scenarios was reduced to multiple sets of binary predictions (true, false) for each scenario. A ROC curve for each loading was computed in a one-vs.-all manner. All other classes are considered negative examples, and only the examined loading was considered positive. This yielded a different ROC curve for each loading. A true positive rate (TPR) was assessed over a false positive rate (FPR) at different thresholds, and the area under the curve (AUC) was calculated. Following Mandrekar (2010), AUC of 0.5 suggested no discrimination, 0.7–0.8 was considered acceptable, 0.8–0.9 was deemed excellent, and larger than 0.9 was considered outstanding. The ROC was calculated for each scenario, and the results were averaged to calculate a macro average (mac). Furthermore, a prevalence-weighted micro average (mic) was calculated treating data as aggregated results. These averages describe the overall performance of the multiclass classification (Asch, 2013). Sensitivity, specificity, and accuracy were calculated based on the mac, where a common threshold was applied.

#### Subject-Specific Load in the Mouse Caudal Vertebra *in vivo*

Mechanoregulation-based load estimation and load history algorithms were applied to the processed longitudinal micro-CT scans. The resulting forces and moments act on different scales and are not directly comparable in magnitude. However, their resulting strain distributions may help understand their impact on tissue scale. In contrast to the *in silico* data, in the *in vivo* data, no ground truth was available to validate the results directly. For the animal data, an anticipated SED distribution was derived based on the experimental assumptions in order to conditionally validate the MR algorithm. The loaded group was subject to an 8 N cyclic load; consequently, a local reference SED distribution was derived for an 8 N load for the loaded group. In accordance with Christen et al. (2012), a 4 N compressive load was assumed for unloaded animals, and the associated SED distribution was derived. The error between LH’s and MR’s load distributions to the reference distributions was calculated for each voxel by subtracting the target’s estimated distribution for each subject at each time point. Voxels were binned according to derived remodelling regions, resulting in error distributions for areas of formation, resorption, and quiescence.

The article "Bone Mechanoregulation Allows Subject-Specific Load Estimation Based on Time-Lapsed Micro-CT and HR-pQCT in Vivo" was published in 2021. Journal: Front Bioeng Biotechnol.

#### Local Mechanoregulation *in silico* and *in vivo*

Conditional probability (CP) curves were calculated for the previously identified remodelling events on the bone surface, in accordance to Schulte et al. (2013), to connect the mechanical environment (SED) as estimated by the algorithms with remodelling sites. Load distribution, resulting from the estimated loads, was normalised using the 99th percentile and binned at 1% steps for each remodelling event. Group-wise normalisation and bin-wise normalisation were used to calculate CP curves for each data set (Schulte et al., 2013). A CCR adapted from né Betts et al. (2020) was calculated to summarise mechanoregulation. This CCR measures the fraction of correctly identified remodelling events using the CP curves.

### Statistics

Statistical analysis was performed using Python 3.8.0, NumPy 1.19.2, and SciPy 1.5.3. Data were tested using an omnibus test of normality based on D’Agostino (1971) and D’Agostino and Pearson (1973) that combines skew and kurtosis. Non-normal parameters were presented as median ± 95% confidence interval (CI) and compared using nonparametric tests: the Wilcoxon–Mann–Whitney test was used for independent and the Wilcoxon signed rank test was used for matched samples. To measure the association between MR and LH predictions and their correlation with grip strength, linear regression analysis was performed; for non-normal parameters, Spearman’s rank-order correlation coefficients were computed to assess the relationship between variables. Normal parameters were presented as mean ± 95% CI and compared using parametric methods: the Student’s *t*-test was used for independent samples, and a paired *t*-test was used for matched samples. For linear regression analysis of normal parameters, Pearson product-moment correlation coefficients were computed. Holm–Bonferroni correction was used for multiple comparisons to reduce the possibility of a type I error. For all tests, a *p*-value smaller than 0.05 was regarded statistically significant. Otherwise, significance levels are reported.

## Results

### Generation of Adapted Bone Geometries *in silico*

For the *in silico* experiments, the goal was to generate adapted bone geometries with constant remodelling rates and known mechanical loads to benchmark the algorithms. The *in silico*-applied force magnitudes were varied until homeostatic remodelling was achieved, resulting in forces between 100 and 600 N. Average BV/TV of the baseline trabecular geometries was 0.12 ± 0.06 and increased to 0.13 ± 0.06 at step 40. An initial drop in BV/TV was observed within the first eight steps of the simulation’s initialisation period and was excluded from further analysis. The temporal resolution between the resulting advection steps needed to be reduced to achieve physiological and constant remodelling rates comparable to *in vivo* follow-up periods. Linear regression analysis showed a significant negative correlation (*R*^2^ = 0.97, *p* < 0.01) between remodelling rates and Pearson’s R between two subsequent images. Hence, Pearson’s R was regarded as a reliable subsampling criterion. Time points were included when a threshold of 0.95 was reached between images resulting in six to eight scans for each geometry and loading scenario. The last six subsampled time points for each experiment and patient were selected for further analysis. This procedure provided highly controlled remodelling rates of 13.79% ± 0.13% between scans.

The article "Bone Mechanoregulation Allows Subject-Specific Load Estimation Based on Time-Lapsed Micro-CT and HR-pQCT in Vivo" was published in 2021. Journal: Front Bioeng Biotechnol.

### Sensitivity, Specificity, and Accuracy *in silico*

A multiclass ROC analysis was used to assess sensitivity, specificity, and accuracy. Average AUCs were high for MR calculated using micro (AUC = 0.98) and macro (AUC = 0.97) averaging. This high value was due to an outstanding performance when classifying uniaxial loads (AUC = 1) (Table 1) and dropped for multiaxial loading cases (AUC = 0.91). An overshadowing of the shear component by compression was observed for CS, resulting in a considerable AUC drop (Table 1). Still, MR exceeded the performance of LH in all categories (Figure 4). Overall, LH only resulted in acceptable micro (AUC = 0.61) and macro (AUC = 0.73) averages, and a below random prediction (AUC = 0.45) was observed for the 6DoF load case. Overall, AUC improved for the calibrated implementation for macro (AUC = 0.79) and micro (AUC = 0.71) averages; however, it was not consistently higher in all categories. At the optimal macro-averaged ROC cut point, load configurations were correctly identified with a high sensitivity of MR. Additionally, the ratio of correctly identified mismatches manifested in high specificity, resulting in an outstanding overall accuracy of MR (Figure 4, upper left panel). In comparison, sensitivity, specificity, and accuracy of LH were significantly lower (*p <* 0.01), yielding only an acceptable differentiation between the applied loading. The calibrated implementation of LH did not achieve significantly higher accuracy compared to the native LH approach and was not further investigated.

The article "Bone Mechanoregulation Allows Subject-Specific Load Estimation Based on Time-Lapsed Micro-CT and HR-pQCT in Vivo" was published in 2021. Journal: Front Bioeng Biotechnol.

**TABLE 1:** Receiver operating characteristic (ROC) derived area under the curve (AUC) for mechanoregulation-based load estimation (MR), load history (LH), and calibrated LH (Cal. LH) for uniaxial loading cases and multiaxial loading.

	Uniaxial						Multiaxial			Average	
	C	SX	SY	T	BX	BY	CS	CB	6DoF	Micro	Macro
MR	0.98	1	1	1	1	1	0.82	0.98	0.93	0.98	0.97
LH	0.83	0.81	0.83	0.71	0.70	0.68	0.69	0.82	0.45	0.61	0.73
Cal. LH	0.87	0.74	0.85	0.96	0.78	0.75	0.66	0.82	0.66	0.71	0.79

*Averages were calculated based on aggregated averaging (macro) and a prevalence-weighted average (micro). C, compressive force in the axial direction; SX, lateral shear force; SY, dorsal shear force; BX, lateral bending moment; BY, dorsal bending moment; CS, combined compression and shear; CB, combined compression and bending; 6DoF, 6-degree freedom load*

**FIGURE 4:** Classification accuracy and ROC for load estimation. Loads of *in silico*-adapted bone geometries (*n* = 5) with nine different loading boundary conditions were estimated and compared to the simulated target load serving as ground truth. Accuracy, sensitivity, and specificity for estimated optimal thresholds were calculated (upper left). Bars show mean, and error bars show 95% confidence interval. All differences between means with *p* < 0.05 are indicated (^∗∗^*p* < 0.01; ^****^p < 0.0001; two-tailed paired *t*-test). Thresholds were derived from multiclass receiver operating characteristic (ROC) for mechanoregulation-based load estimation (MR, upper right), load history LH (lower left), and calibrated LH (lower right).

### Association Between Different Load Estimation Algorithms *in silico*

Linear regression between MR and the target load of the nine *in silico* loading experiments resulted in α_target_ = 1.28 *α_MR_ + 2.64 (*R* = 0.83, *p* < 0.05), slightly underestimating loading magnitude. In comparison, LH showed a weaker correlation and overestimated loads (α_target_ = 0.86 *α_MO_ – 1.80, *R* = 0.45, *p* < 0.05). The calibrated version of LH showed a slightly higher correlation; however, loading magnitudes were underestimated by orders of magnitude indicating that the calibrated version of LH should only be used in combination with a valid calibration equation (α_target_ = 8.36 *α_calMO_ + 36.18, *R* = 0.5, *p* < 0.05).

### Subject-Specific Load in the Mouse Caudal Vertebra *in vivo*

One animal of the loaded group was excluded from the analysis due to convergence issues during the FE analysis. The axial compressive force was predicted as the most dominant loading component for all time intervals using MR (loaded 6.11 ± 1.15 N, control 4.40 ± 1.37 N). Estimations in the loaded group were consistently higher compared to those in the unloaded group (3.73 ± 2.13 N), reaching significantly (*p* < 0.05) higher levels after 2 weeks (Figure 5A). In comparison, the estimations of the axial compressive force by LH only reflected the experimental conditions in the loaded group after the 2-week time point, predicting 5.24 ± 1.42 N in control and 6.40 ± 3.72 N in the loaded group. Using MR, a non-negligible M_x_ moment was predicted in both the loaded (3.97 ± 4.00 Nmm) and control (3.17 ± 1.03 Nmm) groups. Notably high bending moments (> 4 Nmm) in the loaded group were only observed for individual mice, causing large CIs in the predicted M_*x*_ component of the loaded group. In comparison, M_z_ was the largest moment load component indicated by LH for loaded (13.41 ± 0.51 Nmm) and control (14.97 ± 0.33 Nmm) groups and was significantly (*p* < 0.05) higher compared to M_z_ indicated by MR in the loaded (1.41 ± 0.58 Nmm) and control (4.56 ± 1.04 Nmm) groups. Errors for loading estimated by MR were normally distributed (Figure 5B). In comparison, errors for loading estimated by LH were skewed left in regions of resorption resulting in a systematic overestimation of strain in these areas (Figure 5C), indicating a bias of the LH model. Additionally, mean absolute error was significantly (*p* < 0.01) smaller for estimations by MR (f: 0.0051 ± 10^–5^ MPa, q: 0.0057 ± 10^–5^ MPa, r: 0.0042 ± 10^–5^ MPa) compared to LH (f: 0.0071 ± 10^–5^ MPa, q: 0.0070 ± 10^–5^ MPa, r: 0.0081 ± 10^–5^ MPa).

The article "Bone Mechanoregulation Allows Subject-Specific Load Estimation Based on Time-Lapsed Micro-CT and HR-pQCT in Vivo" was published in 2021. Journal: Front Bioeng Biotechnol.

**FIGURE 5:** Load components and error as predicted by mechanoregulation-based load estimation (MR; solid) and load history (LH; dashed) for mouse caudal vertebra (*n* = 8) subjected to physiological (Contr) and extra-physiological loading (Loaded). Bar plots in panel **A** show mean predicted load and standard error (SE) for each component of a 6DoF. Significant differences in prediction between MR and LH with *p* < 0.05 are indicated (^∗^*p* < 0.05; Mann–Whitney–Wilcoxon, Bonferroni). By MR and LH, predicted strain energy density (SED) distributions were compared to an anticipated target load case and distribution was derived from the experimental conditions (contr: 4 N in Fz, loaded: 8 N in Fz). Local error distribution was assessed between estimated and target SED for MR **(B)** and LH **(C)** and grouped in regions of formation, resorption, and quiescence, as derived from time-lapsed micro-CT images. Histograms were truncated at the 98th percentile SED error.

The article "Bone Mechanoregulation Allows Subject-Specific Load Estimation Based on Time-Lapsed Micro-CT and HR-pQCT in Vivo" was published in 2021. Journal: Front Bioeng Biotechnol.

### Patient-Specific Load in the Human Distal Radius *in vivo*

Compressive force, F_z_, was the largest loading component compared to the other unit load cases in the distal radii using both MR (F_z_ = 0.43 ± 0.33 kN) and LH (F_z_ = 0.42 ± 0.27 kN); however, F_z_ did not reach a significantly higher magnitude than F_x_ (0.14 ± 0.09 kN) or F_y_ (0.28 ± 0.13 kN) (Figure 6A). This may be attributed to the large variations in F_z_ predicted by MR and LH across subjects. Mean estimated F_z_ was in good agreement between LH and MR. Using MR, estimated loading was consistent over the 12-month interval, showing no significant difference between time points. Loads estimated using MR showed more considerable variation than LH, which may be due to registration artefacts or variations in image quality between time points.

**FIGURE 6:** Load as predicted by mechanoregulation-based load estimation(MR; solid) and load history (LH; dashed) of physiological load in the human distal radius (*n* = 7). In panel **A**, line plots show mean predicted load and 95% confidence intervals for each component of a six-degree freedom load. No significant differences were found between MR and LH (*p* < 0.05, paired *t*-test). Linear regressions between grip strength and total force ΣF_*i*_ and moment ΣM_*i*_ as predicted by MR **(B)** and LH **(C)** were calculated. Significant correlations indicated (^∗^*p* < 0.05; ^****^p < 0.0001).

Grip strength of individuals was assessed to investigate these variations in compressive force between subjects. Simple linear regression was calculated to predict loads estimated by MR (moment M in Nm and force F in kN) based on grip strength G in kN (Figure 6B). For F, a significant regression equation (F[G] = 3.22 * G - 0.30) was found (*p* < 0.01) with *R*^2^ = 0.72. This correlation between grip strength and forces in the distal radius has been found before and may explain variations among subjects as F increased 3.22 kN for each kN of grip strength. For M, a significant regression equation (M[G] = 0.77 * G + 0.15) was found (*p* = 0.01) with *R*^2^ = 0.18. As such, moment load in the distal radius was less associated with grip strength compared to forces. Simple linear regression for loads estimated by LH reflected a similar trend with a slightly weaker association (Figure 6C). For F, a significant regression equation (F[G] = 2.61 * G - 0.16) was found (*p* < 0.01) with *R*^2^ = 0.70. For M, a significant regression equation (M[G] = 0.26 * G + 0.11) was found (*p* = 0.03) with *R*^2^ = 0.14. A lower correlation between F_*z*_ and grip strength was found for MR and LH.

### Local Mechanoregulation *in silico* and *in vivo*

Mechanoregulation analysis of MR and LH was conducted between subsequent time points for subjects *in vivo* and *in silico* and compared to the results of a commonly used simple compression FE analysis (SC). SED distributions were normalised using the 99th percentile resulting in median normalisation values of 0.071 ± 0.06 MPa for MR, 0.04 ± 0.01 MPa for LH, and 5.28 * 10^–7^ ± 0.01 MPa for SC. Mechanoregulation curves (Figure 7A) showed systematic bone remodelling behaviour, where bone was most likely to be formed in high SED regions, quiescent in medium SED areas, and resorbed in regions of low SED as visually indicated in Figure 8. The *in silico* model’s purely mechanically driven gaussian process was only fully recovered using MR. This anticipated distribution can be seen in the lower-left panel of Figure 7A, showing models generated and analysed using the same SC boundary condition. In comparison, LH’s cp indicated an unphysiological change in curvature localised just above 50% strain.

The article "Bone Mechanoregulation Allows Subject-Specific Load Estimation Based on Time-Lapsed Micro-CT and HR-pQCT in Vivo" was published in 2021. Journal: Front Bioeng Biotechnol.

**FIGURE 7:** Conditional remodelling probabilities (CPs) connecting the mechanical environment [strain energy density (SED)] as estimated by mechanoregulation-based load estimation (MR), load history (LH), and simple compression (SC) with remodelling sites for SC, *in silico* loading (IS), *in vivo* vertebra (CV), and distal radius (DR) datasets. Normalised SED distributions were used to calculate the CP **(A)** for events of formation, quiescence, and resorption to occur at distinct strain levels. Remodelling sites as predicted by the estimated SED were compared to the ground truth, and a correct classification rate (CCR) for *in silico* data **(B)** and *in vivo* data **(C)** was calculated. Boxplots indicate the median and interquartile range. Observations outside the 9–91 scope plotted as outliers. Differences in prediction within and between groups with *p* < 0.05 are indicated (^∗∗^*p* < 0.001; ^****^p < 0.0001; ns *p* > 0.05, two-tailed paired *t*-test within groups, two-tailed individual *t*-test between groups).

**FIGURE 8:** Comparison of remodelling sites with the mechanical environment. Longitudinal *in vivo* high-resolution peripheral quantitative computed tomography (HR-pQCT) scans identified bone formation, quiescence, and resorption and were directly compared to the local mechanical environment. The inset shows an enlarged view of the correspondence between bone formation and high signal and low signal resorption.

To quantify the overall remodelling behaviour, CCR was calculated, measuring correctly classified remodelling events. CCR was significantly higher in the *in silico* data (Figure 7B) than *in vivo* data (*p* < 0.01) as seen in Figure 7C. For the *in silico* data, MR achieved significantly higher CCR (CCR = 0.81) compared to LH (CCR = 0.55, *p* < 0.01). Comparison between the SC (CCR = 0.80) benchmark and MR (CCR = 0.81) showed no significant differences, demonstrating high *in silico* performance of MR. Within the *in vivo* mouse data, no significant differences in CCR were found in the unloaded group (CCR = 0.40) between approaches. However, in the loaded group, CCR predicted using MR (CCR = 0.43) was significantly higher compared to LH (CCR = 0.40, *p* < 0.01) and significantly higher compared to the unloaded group. Finally, within the human distal radius, significantly larger association was found between strain derived from MR (CCR = 0.42) compared to LH (CCR = 0.38, *p* < 0.01) and a higher trend compared to SC (CCR = 0.41).

The article "Bone Mechanoregulation Allows Subject-Specific Load Estimation Based on Time-Lapsed Micro-CT and HR-pQCT in Vivo" was published in 2021. Journal: Front Bioeng Biotechnol.

## Discussion

With the increasing prevalence of bone mechanoregulation studies, this work aimed to extend a previously developed load estimation algorithm (LH) (Christen et al., 2012) by allowing for tissue strain inhomogeneities in our mechanoregulated load estimation approach (MR). These localised differences in mechanical signal may drive bone’s remodelling response and help understand bone mechanoregulation. We provided validation for both algorithms using *in silico*-generated data, *in vivo* HR-pQCT images in humans, and micro-CT images in mice. These experiments indicate the portion of bone remodelling that can be attributed purely to mechanics and establish a baseline for futures studies evaluating mechanoregulation in patients.

Importantly, a combined *in silico* validation and *in vivo* verification, as shown in this study, has not yet been carried out. As such, algorithmic performance quantification was able to be carried out in human radius geometries and mice. Previous studies provided validation using *in vivo* mouse loading experiments (Christen et al., 2012). However, this did not enable the demonstration of algorithmic functionality for load directions other than uniaxial compression, such as those observed in the human distal radius and the mouse vertebra. The consistent results between our *in silico* and *in vivo* loading experiments indicate the validity of the MR algorithmic assumptions under diverse loading conditions. Corroborating the necessity for algorithmic validation in all six degrees of freedom, our *in silico* experiments identified possible performance deficits when applied to complex loading regimes. Despite using the inverse mechanoregulation rules of the advection simulation, MR’s *in silico* accuracy was not perfect for several reasons. First, only six selected time points (out of 40 simulated remodelling steps) were used to generate an *in silico* HR-pQCT scan series that reflected our *in vivo* data. Consequently, the inverse optimisation was challenged to recover loading from an iteratively adapted structure in a single step. Second, the advection simulation’s force-controlled setup caused slight differences in remodelling rates due to the initial anisotropy of the physiological load-adapted bone structure. Here, CS resulted in slightly higher average SED and BV/TV values by favouring bone formation compared to other load scenarios. In contrast to MR, the advection model limits the maximum bone formation rates, which may partially explain the performance deficits within this group.

The article "Bone Mechanoregulation Allows Subject-Specific Load Estimation Based on Time-Lapsed Micro-CT and HR-pQCT in Vivo" was published in 2021. Journal: Front Bioeng Biotechnol.

Although MR’s performance was excellent for simulated adaptation, *in vivo* bone remodelling is not purely load-driven. Predicted *in vivo* loading patterns in the mouse model were in good agreement with a previous study (Christen et al., 2012). Compared to the dataset used by Christen et al. (2012), our LH results showed slightly larger moments while MR predictions were overall in good agreement with the previous study. Our LH results suggest a sizeable torsional component was induced in the caudal vertebra during daily activity, conflicting with the fact that the intervertebral discs limit the transmission of axial moments. Following the model proposed by Schulte et al. (2013), the intervertebral discs of the mouse FE analysis were modelled as stiff tissue (14.8 GPa), which may have resulted in slightly more uniaxial loading. The torsional moment may be affected by this assumption combined with the homogeneous strain simplification of LH as it was not detected using MR. LH-predicted *in vivo* forces in the distal radius model were consistent with a previous study (Christen et al., 2013); however, predicted moments varied by order of magnitude. Christen et al. (2013) used layers of soft-tissue padding at the proximal and distal ends, which may have resulted in further homogenisation of the strains throughout the radius. As such, this step may have limited the transmission of moment load at the interface between calcified tissue and soft tissue. When comparing our results with a cadaveric study investigating distal radius load during various wrist motions (Smith et al., 2018), we find similar load-to-moment ratios, indicating that additional padding may lead to an overestimation of momentum load. Finally, processes such as calcium homeostasis, wherein random bone remodelling may occur, will influence MR estimations. However, the findings of our mechanoregulation analysis reveal that the strain patterns overlap with the pattern observed by natural bone remodelling activity and can be used to estimate *in vivo* loading through our MR reverse engineering approach.

The article "Bone Mechanoregulation Allows Subject-Specific Load Estimation Based on Time-Lapsed Micro-CT and HR-pQCT in Vivo" was published in 2021. Journal: Front Bioeng Biotechnol.

Our data also suggest that estimates in the distal radius may vastly vary from patient to patient. Despite the variance, an increase in loading was associated with increases in grip strength among patients. Such a relationship has been previously reported in cadaveric studies correlating grip strength with joint forces. In agreement with our results, models showed that approximately 26.3 N of force needs to be transmitted through the radius to obtain 10 N of grip strength (Putnam et al., 2000). Although this correlation was significant for loads estimated by MR and LH in the current study, this relationship was largely driven by single individuals with high grip strength. For future distal radius studies, grip strength should be considered as an inclusion parameter. Overall, our results indicate that the internal loads estimated by MR and LH are in good agreement with previous studies and can be linked to external factors such as grip strength in patients.

The principal algorithmic differences between approaches establish different future applications for LH and MR. MR prioritises remodelling sites, which are derived from two subsequent time-lapsed images. Accordingly, MR’s estimation is limited to the time frame between scans. LH estimates loading based on the bone morphology and is therby a cumulative estimate of all prior loadings (load history). Loading during immobilisation treatment (Lill et al., 2003; Clayton et al., 2009; Spanswick et al., 2021), exercise (Troy et al., 2020), or loading interventions (Hughes et al., 2018) may differ from a patient’s load history, which is defined by everyday and occupational activities. Thus, cumulative estimates of LH may be biased by the initial conditions. We showed that initial calibration of LH tends to improve differentiation between loading scenarios; however, this does not allow LH to achieve the same performance as MR. For the mouse loading experiment, this was evident in the delayed detection of significant differences between the loaded and control groups using LH compared to MR. For the present distal radius dataset, patients were skeletally mature adults and did not participate in a specific loading intervention. As a result, there was good agreement between MR and LH estimates. Note that the intact, contralateral radii used in the present study were taken from a patient cohort that had experienced a distal radius fracture. As such, loading in the unfractured arm may have increased, particularly in cases involving fracture of the dominant arm. The resulting change in day-to-day loading may explain slightly higher predictions of MR compared to LH throughout the study. While our results indicate that MR is more sensitive to changes in loading, the algorithm is also more affected by imaging bias than LH. By utilising two subsequent HR-pQCT images, MR is subject to higher noise levels, movement artefacts, and registration errors compared to LH (MacNeil and Boyd, 2008; Sode et al., 2011). LH may be more suited to mouse studies, which can assess lifetime changes, but not for the time frame of most clinical studies of antiresorptive therapies that often assess changes in BMD over a study duration of less than 2 years (Chen and Sambrook, 2012). Overall, our results have confirmed MR’s and LH’s capabilities for various applications using well-defined *in silico* loading and controlled experimental conditions. Accordingly, MR should be used when investigating designated time intervals in a longitudinal analysis and LH to assess the loading history in a cross-sectional fashion or when confronted with low image quality.

The article "Bone Mechanoregulation Allows Subject-Specific Load Estimation Based on Time-Lapsed Micro-CT and HR-pQCT in Vivo" was published in 2021. Journal: Front Bioeng Biotechnol.

To quantify mechanoregulation, we have used a CCR similar to the approach described by né Betts et al. (2020). Here, we show that by using the boundary condition derived by MR, we achieve significantly higher CCR values than LH for simulated, physiological, and extra-physiological loading. Furthermore, our results indicate that these differences are more pronounced when an extra-physiological load was induced. Our results also show that using the simplified compressive boundary condition may be an acceptable choice when investigating trabecular bone mechanoregulation of the healthy human distal radius. However, Johnson and Troy (2018) have shown that this simplified compression boundary condition may alter cortical and trabecular loading sharing. Therefore, the authors caution that such a simplified boundary condition may not be adequate for future studies investigating cortical and trabecular bone mechanoregulation. Although our results indicate a higher trend in CCR for loads estimated by MR, we cannot entirely rule out the possibility that inherent parallels between mechanoregulation analysis and MR synthetically inflate CCR within human distal radius data. However, our analysis of an *in vivo* loading model has provided experimental ground truth showing that estimations by MR reflected experimental conditions properly in mice. Furthermore, our *in silico* validation showed that MR is highly sensitive, specific, and accurate. Overall, our results indicate that mechanoregulation tends to be higher when analysing physiological loading derived by MR and thrives on a wealth of extra-physiological loading. Interestingly, our results also show that simple compression is an adequate simplification for the *in vivo* loading environment in the distal radius considering current limitations. Furthermore, the results of our mechanoregulation analysis revealed a pronounced positive correlation between bone resorption and low strains for our mouse and a human model. This is in agreement with a previous study by né Betts et al. (2020) investigating mechanoregulation in a rodent femoral defect model, which indicated that mechanoregulated bone resorption mainly occurred within the distal and proximal fragments early during recovery. This relationship would indicate that osteoclastic activity may be more sensitive to local strain, and mechanoregulation may differ locally throughout the bone.

The article "Bone Mechanoregulation Allows Subject-Specific Load Estimation Based on Time-Lapsed Micro-CT and HR-pQCT in Vivo" was published in 2021. Journal: Front Bioeng Biotechnol.

The proposed MR algorithm is subject to several limitations attributable to model assumptions as well as experimental and computational constraints. The performed multiclass ROC analysis weighted percent deviations in loading between forces and moments expressed as a reference force, equally. Where forces and moments may have a different impact on tissue level SED, the underlying *in silico* experiments (C, SX, SY, MZ, BX, BY, CS, CB, and 6DoF) were performed at equal loading magnitudes for each geometry, making this method a reasonable *in silico* performance measure. Regarding the animal experiments, the adjacent vertebra’s pinning procedure is limited in precision, and vibrations during the vertebra loading may create slight variations in loading direction and explain the observed higher variability in lateral bending. However, our results are comparable to a previous study (Christen et al., 2012) and represent the experimental setup sufficiently to provide validation for MR and LH. Regarding computational aspects, the method used to determine remodelling sites may include artefacts from scanning, such as beam hardening, motion artefacts, and partial volume effects or numerical inaccuracies of the image registration. However, *in vivo* micro-CT and HRp-QCT have been shown to have sufficient reproducibility for longitudinal bone structure assessment (Ellouz et al., 2014; Scheuren et al., 2020a). Additionally, MR used a Nelder–Mead optimiser that is not a true global optimisation algorithm and may converge in a local solution. However, in practise, it tends to work reasonably well for nonlinear, multimodal, inherently noisy functions. To further counteract this effect, we initialised the optimiser using a least-squares solution (as derived by LH). Future studies confronted with lower image quality may consider using Bayesian Global Optimisation techniques, which come at a higher computational cost but exhibit statistical methods, to address this problem. According to previous work, SED was used as a mechanical signal (Christen et al., 2012, 2013, 2014). More recent studies (né Betts et al., 2020; Malhotra et al., 2021) have identified an effective strain as a preferred candidate for bone mechanoregulation analysis using multi-density FE analysis. However, previous research has shown that these signals are strongly correlated (Pistoia et al., 2002; Ruimerman et al., 2005). Also, the FE model used was linear regarding material and geometry, and load cases were scaled and superimposed linearly during the optimisation to model the compounded loading effect. These simplifications would not capture any nonlinear behaviour or viscoelastic effects; however, only small linear-elastic deformations are expected to occur during day-to-day activity. Future studies may expand this model with increasing computational power and investigate nonlinear effects above yield strength that lead to bone failure (Schwiedrzik and Zysset, 2015).

The article "Bone Mechanoregulation Allows Subject-Specific Load Estimation Based on Time-Lapsed Micro-CT and HR-pQCT in Vivo" was published in 2021. Journal: Front Bioeng Biotechnol.

## Conclusion

We have shown that MR is an enhanced load estimation algorithm tailored for longitudinal bone remodelling studies, achieving high sensitivity, specificity, and accuracy *in silico* by employing acknowledged mechanoregulation principles. The combined *in silico* validation and *in vivo* verification approach presented in this study proved to be a powerful benchmarking tool for the development of time-lapsed bone imaging analysis methods. Moreover, our results indicate that future studies may use grip strength as a functional surrogate to verify estimated patient-specific physiological distal radius loads. Finally, our mechanoregulation analysis revealed considerable amounts of mechanically driven remodelling activity driven in human bone that may enable future studies to understand osteodegenerative disease.

## Data Availability Statement

The raw data supporting the conclusions of this article will be made available by the authors, without undue reservation.

## Ethics Statement

The studies involving human participants were reviewed and approved by Medical University of Innsbruck Ethics Committee. The patients/participants provided their written informed consent to participate in this study. The animal study was reviewed and approved by Swiss Federal Food Safety and Veterinary Office.

## Author Contributions

MW, NO, MB, RM, and CC: study design. MW and FM: study conduct. MW and MB: data collection. MW, NO, and FM: data analysis. MW, FM, NO, RM, and CC: data interpretation, revising manuscript content, and approving final version of manuscript. MW and CC: drafting manuscript. CC: takes responsibility for the integrity of the data analysis. All authors contributed to the article and approved the submitted version.

The article "Bone Mechanoregulation Allows Subject-Specific Load Estimation Based on Time-Lapsed Micro-CT and HR-pQCT in Vivo" was published in 2021. Journal: Front Bioeng Biotechnol.

## Conflict of Interest

The authors declare that the research was conducted in the absence of any commercial or financial relationships that could be construed as a potential conflict of interest.
